# Animal Models and Pathogenesis of Ulcerative Colitis

**DOI:** 10.1155/2022/5927384

**Published:** 2022-07-11

**Authors:** Xin Gao, Jia Li, Xueping Pang, Kaiyuan Cong, Chunlei Jiang, Bingxuan Han, Jiawei Gao, Zhihao Wang, Jiangshan Hu, Kaijun Wen, Xinfa Ye, Liwen Dou

**Affiliations:** Shandong University of Traditional Chinese Medicine, Shandong, China

## Abstract

**Background:**

Ulcerative colitis (UC) is a kind of inflammatory bowel disease which is needed to be predicted.

**Objective:**

To analyze various animal models of UC conditions and summarizes the animal selection, model progression, and pathogenic mechanisms of UC animal models.

**Methods:**

We surveyed the research papers published in PubMed, Google Scholar, Baidu Scholar, CNKI, SciFinder, and Web of Science in the past 5 years and discussed the experimental animals, modeling methods, and pathogenic mechanisms.

**Results:**

In the selection of experimental animals, rats are considered the best experimental animals. The mainstream modeling methods can be categorized into the chemical stimulation method, immune stimulation method, and compound method, among which the compound method is the most successful. In the study of the pathogenesis of UC, the pathogenesis of UC is due to various pathogenic factors, such as nitric oxide (NO), prostaglandins (PG), proinflammatory factors (IL, TNF-*α*), and intestinal flora.

**Conclusion:**

The method of building an animal model of UC is well-established, providing a more targeted selection of animal models for future related experiments.

## 1. Introduction

UC is an intractable, cancer-prone, refractory gastrointestinal disease, since Stephen et al. first described the pathology of diseases such as colitis or idiopathic colitis [1]. In recent years, the incidence of the disease has been increasing, and it has been classified as one of the intractable diseases by the World Health Organization (WHO) [2]. Currently, there is no effective treatment for UC, and the current main treatment is also based on controlling the inflammatory response of the intestine and controlling complications. At present, the clinical treatment of this disease mainly uses corticosteroids, aminosalicylic acid preparations, immunomodulators, and other drugs, but the disease has the characteristics of high recurrence rate, and long-term medication can easily lead to the occurrence of adverse reactions. Among them, aminosalicylic acid preparations and glucocorticoids are first-line drugs for the treatment of UC, but due to the complexity of the disease, the cause has not been fully defined, and the clinical efficacy cannot fully meet the needs of patients. With the development of molecular biology, some advancement of treating UC has been made, but how to completely cure this disease is still challenging.

In order to explore the pathogenesis of UC, it is crucial to establish relevant animal models. The development of UC is mainly related to genetic, environmental, gut microbiome, immunity, infection, and psychological aspects [3], which suggests that the onset of UC is the result of multifactorial action. Therefore, UC cannot be completely cured by a single drug or clinical treatment, it has become crucial to explore the pathogenesis of UC through animal models.

Experimental animal models have many advantages in studying the mechanisms of UC development: it can simulate the whole process of UC occurrence and development. Therefore, it became crucial to build a laboratory animal model of UC disease that was highly identical to the human gut environment. However, before building an animal model of UC, the most basic and important thing is the selection of laboratory animals.

In the selection of experimental animals, it should be in line with the following four principles: the use of experimental animals similar to human structure, function, metabolism, and disease; the use of standardized experimental animals; the use of experimental animals with some special reactions, sensitive to stimuli; the use of zoonotic experimental animals; and the use of easily available and economical experimental animals [4].

According to the above principles, we should first choose animals that are suitable for UC disease modeling, closest to the human internal environment and most reflective of clinical drug efficacy. In recent years, rats and mice have been widely used in many animal experiments: they are genetically close to humans, tame and easy to handle, they have good intraperitoneal injection effect, their white body hair is easy to observe, and they are cheap and easy to keep.

However, to choose an animal that best fits the human intestinal environment and is most suitable for investigating UC disease, it is also important to distinguish the differences between rats and mice. On the one hand, mice have a shorter intestine, while rats have a longer intestine, about 114 cm (102-126), and the classification of the rat intestine is similar to that of humans, so rats are superior to mice in this respect; on the other hand, rats are omnivorous, anatomically and physiologically similar to humans, and have a fast growth and metabolism, and rats can be used for nutritional and pharmacological studies. In addition, rats are also the main experimental animals for drug evaluation and can be made into animal models of experimentally induced genetic defects diseases similar to those of humans. These advantages are very beneficial for modeling UC diseases, whereas mice do not have a significant advantage in modeling UC, so rats are more preferred for modeling.

If an animal model of UC that fits the human intestinal tract can be successfully established, various experiments can be conducted based on this model to test the therapeutic effects of various clinical drugs on UC as well as further analyze the pathogenesis of UC. Eventually, we may be able to come up with a set of treatment plan to cure UC through the in-depth study of this model.

By the in-depth comparative analysis of various animal models of UC conditions, this paper summarizes the animal selection, model progression, and pathogenic mechanisms of UC animal models and provides a more targeted selection of animal models for future related experiments. We surveyed the research papers published in PubMed, Google Scholar, Baidu Scholar, CNKI, SciFinder, and Web of Science in the past 5 years and discussed the experimental animals, modeling methods, and pathogenic mechanisms.

The rest of the manuscript is arranged according to the following agenda items where a brief description of every section is provided. In Section 2, the proposed mechanism, i.e., methodology which is reported in the paper, is described in detail. In Section 3, various results of the proposed scheme were described in detailed along with description of the efficacy of the proposed methods in resolving the issue under consideration in this paper. Finally, concluding remarks are given.

## 2. Proposed Methodology

We surveyed papers related to UC research published in PubMed, Google Scholar, Baidu Scholar, CNKI, SciFinder, and Web of Science over the past 5 years and searched for UC-related conference papers and studies related to UC in obsolete journals. The three investigators screened the UC-related literature, assessed the quality, extracted basic information, participants (animals or humans), intervention protocols, outcome measures (UC-related indicators), relevant progress, and modeling methods. The Cochrane risk assessment tool was employed to evaluate the quality of the literature, and the software RevMan 5.3 and Stata14 were used to conduct the analysis, and finally, the experimental animals (humanoid, standardized, sensitive, zoonotic, economical, and practical), modeling methods (frequent application, high feasibility), and pathogenic mechanisms (comprehensiveness, focus, and credibility) were summarized and analyzed, as shown in Table 1.

## 3. Evolution of the Modeling Methods

Modeling methods of UC used in the last 30 years, as shown in Table 2.

Figure 1 shows the evolution of UC modeling methods and the general trend of their evolution. Before the 21st century, most of the modeling methods such as immunostimulation were used. In the early 21st century, DNCB (Figure 2) with acetic acid, ethanol enema, and TNBS (Figure 3) ethanol enema became the commonly used methods. After 2014, DSS induction methods became prevalent; sometimes, it is combined with DMH (Figure 4). In the last 30 years, colonic transplantation and oxazolone (OXZ) modeling methods have also emerged, but they are used less frequently. It has been found that most of the modeling methods are still commonly used by the composite method and chemical stimulation method (Figure 5), with the composite method being more accurate. The composite method uses multiple reagents to perform the modeling, which avoids the disadvantages of long modeling time and short duration of disease due to single reagent modeling, and greatly improves the success rate and reproducibility of modeling.

## 4. Pathogenesis

### 4.1. Pathogenic Factors

The causes of UC pathogenesis are not clearl yet. Dietary habits, psychological factors, and lifestyle habits play an important role in the deterioration of the disease, and genetic factors may also lead to the UC. In addition, some studies have suggested that UC is an autoimmune disease [58].

In terms of dietary habits, behaviors such as overeating, consuming fried, high cholesterol, high sugar, and high protein foods, lack of attention to food hygiene, and excessive alcohol consumption can increase the burden on the gastrointestinal tract and decrease the immunity of the gastrointestinal tract, thus increasing the risk of inflammatory bowel disease (IBD) [59]. High intake of sulfur-containing foods also increases the incidence of UC; excessive intake of sulfur-containing foods increases H_2_S levels, which leads to damage to the intestinal mucosal barrier and ultimately increasing the incidence of UC [60–62]. High intake of alcohol can directly cause mucosal damage and increase bacterial translocation, which is a risk factor for UC.

In terms of psychological factors, if the mental state is under high pressure and stressful environment for a long time, the adrenal axis, mucosa, and pathogens will interact and contribute to the activation of mast cell activity in the intestinal mucosa, generating hormones that cause intestinal inflammation and eventually triggering UC [63, 64].

For the lifestyle habits, the usual irregular work and rest, long hours of stressful work, overwork, antiseasonal dressing, and lack of physical exercise may cause a decrease in autoimmunity, which may trigger UC. In addition, fulminant, acute attacks, and severe chronic patients who do not rest in bed may also aggravate the disease.

### 4.2. Pathogenic Factors and Mechanisms

To establish a better animal pathological model of UC, it is necessary to understand the pathogenic factors and mechanisms of action, and only by in-depth investigation can we understand which modeling method is the most suitable. Studies have shown that the presence or absence of pathogenic factors such as nitric oxide (NO), prostaglandins (PG), proinflammatory factors (IL, TNF-*α*), intestinal flora, and their levels may trigger UC pathology, but their mechanisms are different.

#### 4.2.1. Nitric Oxide

NO plays a dual role in the human intestine: small amounts of NO in the body protect the intestinal mucosa while promoting coagulation to form thrombi [65]; while large amounts of NO produced at the onset can damage the intestinal mucosa and damage intestinal tissues. Irritation of the intestinal mucosa of patients at the onset of UC infiltrates granulocytes and oxidative stress (OS) occurs, in which oxygen is electronically reduced to produce superoxide (O_2_·-), and inducible nitric oxide synthase (iNOS) by genetic control [66], synthesizes high levels of NO with O_2_·-. NO acts as a potent inflammatory mediator that inhibits the secretion of immunoreactive substances in the body, and the excessive release of NO leads to increased intestinal increased vascular permeability and promotes secretion of intestinal epithelial cells, causing inflammation, edema, and congestion of the intestinal mucosa, as shown in Figure 6, which clinically manifests as abdominal pain, diarrhea, and bloody stools, along with cytotoxic effects [67].

#### 4.2.2. Prostaglandins

Arachidonic acid (AA) is the main substance for the release of endogenous prostaglandins in the body, while cyclooxygenase (COX) is the key enzyme that catalyzes the production of prostaglandins from AA, and inducible COX (COX-2) is one of the isoenzymes of COX. At the onset of UC, COX-2 is stimulated by pathogenic factors such as NO, which catalyzes the release of large amounts of prostaglandin-like substances from AA. Prostaglandin E_2_ (PGE_2_) (Figure 7), one of the main substances released from AA (Figure 8), is a proinflammatory factor that induces granulocyte infiltration in the intestinal mucosa, thus triggering the oxidative stress process, accompanied by the release of large amounts of NO [68], causing inflammation and edema in the intestinal mucosa, as shown in Figure 6. PGE_2_ also accelerates cell proliferation, thereby inhibiting the immune action of immune T cells [69], causing immune damage and possibly inducing tumorigenesis [70]. It has been demonstrated [71] that the intestinal mucosal damage induced by DSS can be alleviated by inhibiting the COX-2 process.

#### 4.2.3. Proinflammatory Cytokines

Proinflammatory factors in humans are produced by Th1 cells, CD4+ cells, macrophages, and dendritic cells. The main proinflammatory factors produced are IL-1, IL-6, and TNF-*α*. IL-1*β* is produced by activated macrophages and mainly controls the immune inflammatory response in the gut. TNF-*α*, similar to IL-1*β*, is also a pleiotropic proinflammatory cytokine that affects the production and secretion process of multiple inflammatory mediators [72] (Figure 9).

Local activation of IL-1*β* is central in mediating the proinflammatory response, leading to the activation of secondary inflammatory mediators (IL-6); at the same time, IL-6 is considered to be an amplifier of certain biological effects of IL-1*β*, TNF-*α*, etc., which in turn can promote the proinflammatory effect of IL-1*β* and lead to increased inflammation of the intestinal mucosa. IL-6 can also have a cellular effect on B cells, T cells, and other immune cells proliferation and cause immune damage. Studies have shown [73] that IL-1*β* and TNF-*α*, as initiators, regulate pain by altering COX-2 levels. Clinical progress is often determined by monitoring inflammatory levels of serum IL-1*β*, IL-6, and TNF-*α* [74, 75].

#### 4.2.4. Intestinal Flora

There are various types of flora in the human intestine, such as Bacteroidetes, Tenericutes, and Shigella Castellani of E. coli [76]. When the organism operates normally, the number of various flora is kept in a certain balance. However, if the balance of the normal number of flora is disrupted, it will lead to a decrease in the biodiversity of the flora in the human body, with a decrease in beneficial genera and an increase in harmful genera. The increase of harmful genera may reduce the thickness of the mucus layer and aggravate the damage of the intestinal mucosal barrier [77], thus inducing intestinal inflammation. Among them, diffusely adherent E. coli can initiate their interaction with fully differentiated epithelial cells through bacterial recognition of decay/acceleration factor (DAF), carcinoembryonic antigen-associated cell adhesion molecule CEACAM1 or CEACAM6 [78] (Figure 10), as shown in Table 3, which ultimately leads to the development of intestinal inflammation.

## 5. Classification of Modeling Methods and Their Pros/Cons

An in-depth investigation of modeling approaches in the last 5 years of UC animal models revealed that the main modeling approaches were broadly classified into three categories: chemical stimulation, immunostimulation modeling approaches, and composite approaches. These three types of modeling methods are very different from each other in terms of methods and drugs used and are highly comparable and specific. However, each of these three main categories of modeling methods is subdivided into several different types of modeling methods. In general, the pathogenic factors and virulence factors are generally the same for the same category of modeling approaches, but there are subtle differences in the duration of pathogenicity, duration of disease, and quality of animal models. In the following section, we summarize the specific modeling methods that are currently available for the more successful modeling approaches and their advantages and disadvantages.

### 5.1. Chemical Stimulation Methods

Stimuli are changes in the internal and external environment that can be felt by the body and cause reactions in tissue cells, organs, and the organism. Among them, stimuli triggered by acids, bases, drugs, etc. are chemical stimuli. When the human organism is diseased, some chemical factors in the human body will also change in content and presence or absence. Similarly, changes in the levels of some chemical factors in the human body that are not treated in time can lead to lesions of UC. With this idea, many researchers have used some chemical reagents to stimulate the animal organism to change the level of chemokines in the body to achieve the ultimate success of the model, which is called the chemical stimulation method.

As shown in Table 4, the main chemical drugs used in the chemical stimulation method are as follows:

1. DSS
2. OXZ
3. DNCB
4. TNBS

### 5.2. Immunostimulation Method

Immunity refers to the function of the body's immune system to recognize itself and foreign substances and to exclude antigenic foreign substances through immune response in order to maintain the physiological balance of the body. Immunity is divided into two types: natural immunity and acquired immunity. Natural immunity is inherent to the individual and is generally non-specific, such as the role of phagocytes in the human body. Acquired immunity is divided into automatically acquired immunity and passively acquired immunity. Automatically acquired immunity is generally long-lasting and can last for life, such as measles, smallpox, and mumps. Passive acquired immunity: immunity time is short, artificially acquired with a long time, and has been less used. In the process of establishing animal models of UC, some modeling methods are the same as the process of immunization, the easily sensitized chemical drugs through different methods to stimulate the animal collective, the body after the occurrence of immune response, leading to disruption of the immune system, which triggers the development of UC lesions in the organs of the animal.

Immunostimulation modeling methods can be broadly divided into (see Table 5): (1) colonic mucosal tissue sensitization method, (2) rat colonic bacterial strain method, (3) fetal rat colonic implantation method, and (4) spontaneous animal models.

### 5.3. Composite Method

The composite modeling method is the combination of multiple modeling methods, which summarizes the advantages and defects of various modeling methods and combines them to obtain a better modeling method. Since the composite method is not too complicated and has better pathological restoration, it is now widely used in the construction of UC animal models.

As shown in Table 6, the main chemical combinations currently used in the composite method are as follows:

1. TNBS+ethanol
2. DNCB+acetic acid composite method
3. DNCB+ethanol
4. DSS+acetic acid
5. DNCB+acetic acid+ethanol
6. DMH+DSS

By summarizing the modeling methods of UC animal models used in the existing studies over the past years, we found that most studies still use chemical stimulation method, which is simple, easy to repeat, and easy to recreate; on the contrary, the immune method is usually strict, the success rate of final modeling is low, and the time and capital costs are too high, so it is less used at present; the compound method is more flexible, which can focus on different research directions in modeling according to the different needs of multiple UC animal models, and the frequency of the compound method is gradually increasing in recent years.

## 6. Results and Discussion

### 6.1. The Animal Selection in Modeling of UC

In the animal modeling of UC, rats are the better experimental animal subjects. We find that there is no uniform requirement for the selection of experimental animal models for UC. Rats are the most reliable experimental animal model for UC because they are easy to obtain and similar to the human intestinal system and rich experimental data has been produced.

### 6.2. The Modeling Method of UC

Among the mainstream modeling methods in UC research, the composite method is the most successful. In the 20th century, most experimental studies on UC used immunostimulation for modeling. These experiments were less carried out, the experiments lacked credibility and these experimental methods were more complex and cumbersome. After 2000, the compound method and chemical stimulation method were gradually developed in UC animal modeling, in which the operation of the compound method is simpler, only need to establish animal models and index testing to obtain the corresponding animal experimental results, and only need to use some reagents such as 0.1% DNCB and acetic acid in the establishment of animal models. The reagents are convenient and effective, so the compound method is the most successful in UC modeling.

### 6.3. The Pathogenesis of UC

In the pathogenesis of UC, it may be influenced by various pathogenic factors and pathogenic factors. Existing studies clearly suggest that UC is a group of chronic nonspecific inflammatory diseases of the colon and rectum. According to the current research, the pathogenesis of UC is still unclear, but with the in-depth research of domestic and foreign scholars, it is found that UC may be related to genetics, immunity, susceptibility genes, and environmental factors [102]. We found that genetic factors play a certain role in the pathogenesis of UC, and psychologically induced factors are also critical in the deterioration of UC.

In chemical measurements, nitric oxide (NO), prostaglandins (PG), and proinflammatory factors (IL, TNF-*α*) are found to play a catalytic role in the pathogenesis of UC; the final outcome of which is the possibility of forming UC or accelerating the progression of UC disease. It is mainly related to immunity: (1) proinflammatory factors (TNF-*α*, IL-1*β*, IL-6, IL-12, and IL-23) and anti-inflammatory factors (IL-2, IL-4, and IL-10) imbalance; (2) regulatory T cell dysregulation, (3) platelet activation, (4) upregulation of leukocyte antigen (HLA), and (5) Increased perinuclear neutrophils [103]. In addition, iron death due to iron deposition has been reported [103, 104] and may be the main underlying mechanism of ulcerative colitis and has been shown to be Nrf2/HO-1 as its pathway. MicroRNAs such as miR-21 and miR-146a are endogenous nonprotein-coding RNAs that play an important role in various stages of cells and are closely related to various stages of UC development, such as maintaining intestinal epithelial function and related pathways affecting inflammatory factors [105, 106]. The pathogenesis of UC has not yet been clearly established, so the establishment of suitable animal models has become an indispensable tool for studying disease mechanisms and developing therapeutic methods. The intestinal part of the human body is host to tens of trillions of bacteria; these strains maintain the balance under specific conditions, allowing the body to maintain a normal healthy state. Once the balance of the flora breaks down, harmful strains dominate, which may also cause damage to the intestinal barrier. Eventually, it leads to the occurrence of intestinal inflammation, and it most likely catalyze the occurrence and development of UC.

## 7. Conclusion and Future Direction

By the in-depth comparative analysis of various animal models of UC conditions, this paper summarizes the animal selection, model progression, and pathogenic mechanisms of UC animal models and provides a more targeted selection of animal models for future related experiments. We surveyed the research papers published in PubMed, Google Scholar, Baidu Scholar, CNKI, SciFinder, and Web of Science in the past 5 years and discussed the experimental animals, modeling methods, and pathogenic mechanisms. In summary, there are various methods for preparing experimental models of UC animals for scientific experiments, among which the immunostimulation method was the first to appear, followed by the chemical stimulation method and the composite modeling method. In the selection of experimental animals, we compared the advantages and disadvantages of various experimental animals for the animal model of UC and finally selected rats as the best experimental animals after combining with the human intestinal physiological environment. The common causative factors of UC, such as prostaglandins, proinflammatory factors, and intestinal flora, also have different mechanisms of action and development.

In future research, the study of the mechanism of UC disease combined with animal models is a key entry point for Chinese and Western medicine to explore the mechanism of treatment of the disease and to develop therapeutic methods. It should be fully integrated with the achievements of modern science, while demonstrating the characteristics of each of the multiple treatment modalities. An ideal animal model can help restore the key mechanisms of colorectal UC development and is crucial for research such as the discovery of new impact factors and the selection of better experimental animals. The above models have their own advantages and disadvantages, but they are only similar to UC in some pathological changes, etc., and it is difficult to become an ideal model for studying UC. The etiology and pathogenesis of UC, especially the immunological mechanism, are very complex and the disease is prolonged. The currently established animal models are difficult to reflect the immunological response and mechanism of human UC. An ideal animal model of IBD should have the following characteristics [103]: (1) Its intestinal inflammatory progression and pathophysiological changes are similar to IBD. (2) Laboratory animals must have a clear genetic background that well reflects the interaction between humans and the intestinal flora. (3) Specific antigens can induce corresponding intestinal immune responses with good reproducibility. (4) Traditional approaches to IBD treatment are effective in the induced model. (5) Intestinal inflammation should be spontaneous and not caused by genetic modification or chemical treatment. A good animal model can facilitate us to explore the etiology, pathogenesis, and efficacy of therapeutic drugs in humans from different perspectives. As most genetically modified spontaneous models, the onset and severity are highly dependent on environmental factors, leading to high variability in studies. Acute and chronic UC models induced by chemical methods, because of their low cost, controllability, and reproducibility, can only reflect a certain aspect of UC but are still the most commonly used methods in UC research. Further investigation and screening are required to explore other more superior animal models of UC and to assess their experimental feasibility and possible interactions with other pathologies. Therefore, in-depth research, integration, and refinement of experimental animal selection, improvement of modeling methods and exploration of pathogenic factors under the current modeling advances will be promising for the preparation of stable and comprehensive UC animal models as well as standardized modeling criteria. There are also a variety of options for how animal models of UC are replicated, but how to choose a safer, more stable animal model that reflects the symptoms of clinical UC patients has always been the focus of research. How to prepare a stable UC TCM animal phenological model and standardized model standards needs to be explored, integrated, and improved.

## Figures and Tables

**Figure 1:** Evolution of UC modeling methods in the last 30 years.

**Figure 2:** Chemical structure of DNCB.

**Figure 3:** Chemical structure of TNBS.

**Figure 4:** Chemical structure of DMH.

**Figure 5:** Chemical structure of DSS.

**Figure 6:** Mechanism of NO and PGE_2_ synergistic action to induce UC.

**Figure 7:** Chemical structure of PGE_2_.

**Figure 8:** Chemical structure of AA.

**Figure 9:** Mechanism of the interleukin factor stimulation of T cells to induce UC.

**Figure 10:** Mechanism of UC induction facilitated by intestinal flora through DAF recognition by DAEC.

**Table 1:** Experimental animals, modeling methods, and principles of pathogenesis.

Category	Principle of selection
Experimental animals	Humanoid, standardized, sensitive, zoonotic, economical, and practical
Modeling method	Frequent application, high feasibility
Pathogenesis	Comprehensiveness, focus, credibility

**Table 2:** Modeling methods of UC used in the last 30 years.

Time	Modeling chemicals	Categorization	References
1990	Human postoperative colonic mucosal supernatant+Fruend adjuvant	Immunostimulation method	[5]
1992	Acetic acid	Chemical stimulation method	[6]
1995	Bacterial suspension made from rat colonic contents	Immunostimulation method	[7]
1995	Dextran sodium sulfate (DSS)	Chemical stimulation method	[8]
1997	Colonic transplantation	Immunostimulation method	[9]
1998	Human postoperative colonic mucosal supernatant+Fruend adjuvant	Immunostimulation method	[10]
1999	Acetic acid	Chemical stimulation method	[11]
1999	Human postoperative colonic mucosal supernatant+Fruend adjuvant	Immunostimulation method	[12]
2000	Human postoperative colonic mucosal supernatant+Fruend adjuvant	Immunostimulation method	[13]
2002	Antigenic emulsifier	Immunostimulation method	[14]
2002	2.4-Dinitrochlorobenzene (DNCB)	Chemical stimulation method	[15]
2002	Trinitrobenzene sulfonic acid (TNBS)+ethanol	Composite method	[16]
2003	Human postoperative colonic mucosal supernatant+Fruend adjuvant	Immunostimulation method	[17]
2003	TNBS+ethanol	Composite method	[18]
2004	Oxazolone (OXZ)+ethanol	Composite method	[19]
2004	Acetic acid	Chemical stimulation method	[19]
2004	DNCB	Chemical stimulation method	[20]
2005	TNBS+ethanol	Composite method	[21]
2005	1.2-Dimethylhydrazine (DMH)+DSS	Composite method	[22]
2005	Acetic acid	Chemical stimulation method	[23]
2005	DNCB+acetic acid	Composite method	[24]
2006	TNBS/DNCB	Composite method	[25]
2006	DNCB+ethanol	Composite method	[26]
2006	TNBS+ethanol	Composite method	[27]
2006	DNCB	Chemical stimulation method	[28]
2007	TNBS+ethanol	Composite method	[29]
2008	DNCB	Chemical stimulation method	[30]
2008	DNCB	Chemical stimulation method	[31]
2008	TNBS	Chemical stimulation method	[32]
2008	DSS	Chemical stimulation method	[33]
2009	DSS+acetic acid	Composite method	[34]
2009	TNBS	Chemical stimulation method	[35]
2010	DSS	Chemical stimulation method	[36]
2011	DMH	Composite method	[37]
2011	TNBS+ethanol	Composite method	[38]
2011	DSS	Chemical stimulation method	[39]
2012	DSS	Chemical stimulation method	[40]
2012	TNBS+ethanol	Composite method	[41]
2013	TNBS+ethanol	Composite method	[42]
2014	TNBS+ethanol	Composite method	[43]
2014	DSS+DMH	Composite method	[44]
2014	DSS	Chemical stimulation method	[45]
2014	DNCB+acetic acid	Composite method	[46]
2015	TNBS	Chemical stimulation method	[47]
2016	DNCB	Chemical stimulation method	[48]
2017	DSS	Chemical stimulation method	[49]
2017	TNBS+ethanol	Composite method	[50]
2018	DSS	Chemical stimulation method	[51]
2019	DSS	Chemical stimulation method	[52]
2019	DNCB+ethanol+acetic acid	Composite method	[53]
2019	TNBS+ethanol	Composite method	[55]
2020	DSS	Chemical stimulation method	[54]
2020	DSS	Chemical stimulation method	[55]
2021	DSS	Chemical stimulation method	[56]
2021	DSS	Chemical stimulation method	[57]

**Table 3:** Pathogenic factors and mechanisms of action of important UC-causing drugs.

Drug name	Pathogenic factor	Mechanisms	Reference
DSS	IL-1, IL-6, TNF-*α*, intestinal flora	Elevated mRNA levels of IL-1, IL-6, TNF-*α*, and secreted levels in serum; dysbiosis of intestinal flora by increasing the permeability of intestinal mucosal cells.	[79] [80]
OXZ	Th1/Th2 cytokines (TNF-*α*, IL-6)	Leading to an imbalance in the ratio of Th1/Th2 helper cells, increased release of TNF-*α* and IL-6, active secretion of B lymphocytes, production of antibodies, and hyperactive humoral immune response, which in turn activates the complement system and causes an inflammatory response in the intestinal mucosa.	[81] [82]
DNCB	NO, TNF-*α*	Activation induced by T cells, resulting in a significant increase in NO and TNF-*α* activity	[83]
TNBS	Intestinal flora, IL-6, TNF-*α*	Elevated IL-6 and TNF-*α*, disrupts the structure and composition of the intestinal flora, causing disruption of the flora.	[84, 85]

**Table 4:** Establishing UC model based on chemical stimulation methods.

Drug name	Modeling method	Animal	Specific modeling method	Advantages	Disadvantages	References
DSS	Free drinking or gavage	Rats	DSS solution free drinking for 7 d or DSS solution by gavage for 7 d.	Easy to make, high success rate, good reproducibility, lesion symptoms are very similar to human UC.	Long modeling period, influenced by many factors, unstable experimental data, difficult to make a successful and stable model.	[86–88]
		Mice	DSS solution free drinking for 7 d or DSS solution by gavage for 7 d.			
OXZ	Skin sensitization+gavage	Rats	Oxazolone applied to exposed skin for 7 d continuously combined with oxazolone gavage.	Simple operation, rapid model establishment, good reproducibility, very similar to UC in humans.	Duration of disease is maintained for a relatively short period of time and the exact mechanism is not fully understood.	[80] [89]
		Mice	Oxazolone ethanol solution combined with oxazolone ethanol solution enema.			
DNCB	Skin sensitization+enema	Rats	DNCB for 7 d, then DNCB, enema for 2 d.	Simple operation, high similarity in pathology to human UC.	More tedious operation, requires prior sensitization, inflammation is self-healing.	[90]
TNBS	Enema	Rats	TNBS ethanol solution enema.	Simple operation, good reproducibility, shorter time to induce ulceration, longer duration of lesions.	TNBS stimulation is too severe, easy mucosal ulceration perforation, and death.	[91] [92]
		Mice	TNBS enema for 7 d.			

**Table 5:** Immunostimulation method UC model.

Name	Modeling method	Animal	Specific modeling method	Advantages	Disadvantages	References
Colonic mucosal tissue sensitization method	Injection+enema	Rats	Injection of antigen-containing Fuchs' antigen emulsion+enema with ethanol solution.	Longer duration of lesions; similar to human UC immunopathogenesis; suitable for screening of new drugs.	Longer modeling time; more cumbersome operation; multiple injections of antigen required to maintain sensitization.	[93]
Rat colonic bacterial strain method	Injection	Rats	Bacterial suspensions were made from E. coli in the colon contents of healthy rats, and the suspensions were injected.	Longer maintenance of inflammation; mostly chronic inflammation.	Longer time required to prepare E. coli suspensions requires certain conditions and techniques.	[7]
Fetal rat colonic embedding method	Surgical embedding	Rats	The fetal rat colonic was removed 3-4 cm long and surgically embedded aseptically under the right kidney pericardium in adult rats.	Animal disease, the disease model is similar to the clinical symptoms of UC.	High technical requirements; long experimental period; low success rate.	[94]
Spontaneous animal models	Abnormal mutations in genes, selective breeding and hybridization	Serratia marcescens	Abnormalities occurring under natural conditions or genetic mutations; obtained by relying on selective breeding and hybridization methods.	The closest model to the occurrence of UC; reflects well on the development of UC and the effect of drug treatment.	Difficult to standardize control; and animals are scarce and expensive, making it difficult to apply to large-scale experiments or more in-depth studies.	[95]
		Mice				

**Table 6:** Composite method to establish UC model.

Name	Modeling method	Animal	Specific modeling method	Advantages	Disadvantages	References
TNBS+ethanol	Enema	Rats	TNBS ethanol solution enema	Modeling method is simple and economical; high modeling efficiency; good model stability; good reproducibility; similar to human UC.	Its inflammatory manifestations are more similar to Crohn's disease.	[96] [28] [97]
		Mice	TNBS ethanol solution by enema, and 7 d later by TNBS ethanol solution by enema.			
DNCB+acetic acid	Skin sensitization+enema	Rats	DNCB acetone solution drip back once for 14 d and enema with DNCB ethanol solution for 15 d.	Consistent with UC characteristics; long duration, high success rate, reproducible and simple.	Modeling is cumbersome.	[98]
DNCB+ethanol	Enema	Rats	DNCB ethanol solution for 2 d continuously	Overcome the short duration and lack of self-healing of DNCB; similar to human UC.	Long time required for modeling.	[53] [99]
	Skin sensitization+enema	Mice	DNCB solution applied to abdomen for 4 d followed by DNCB ethanol solution enema for 5 d.			
DSS+acetic acid	Free drinking+enema	Rats	Free drinking of DSS solution for 7 d, fasting without water for 1 d and enema with acetic acid solution.	Simple and easy to perform; short modeling time; high success rate; good reproducibility; long self-healing time.	Acetic acid enema is likely to cause death in rats.	[100]
DNCB+acetic acid+ethanol	Skin sensitization+enema	Rats	DNCB acetone solution dribbled back for 14 d, enema with DNCB ethanol solution for 15 d, acetic acid solution injected at same site for 16 d.	Similar to human colorectal UC disease.	Acetic acid enema tends to cause animal death.	[101]
DMH+DSS	Intraperitoneal injection+free drinking	Mice	Intraperitoneal injection of DMH and free drinking of DSS, with 18 weeks.	Simple and easy; good reproducibility; similar to human UC disease.	Large doses or prolonged use of DMH can induce intestinal cancer.	[44]

## Data Availability

The datasets used and analyzed during the current study are available from the corresponding author upon reasonable request.
